The article "A follow-up study of children with posterior urethral valve" was published in 2010. Journal: Indian J Nephrol.

# A follow-up study of children with posterior urethral valve

**DOI:** 10.4103/0971-4065.65298

**Published:** 2010-04

**Authors:** S. Uthup, R. Binitha, S. Geetha, R. Hema, L. Kailas

**Affiliations:** SAT Hospital, Government Medical College, Thiruvananthapuram, India

**Keywords:** Chronic kidney disease, glomerular filtration rate, posterior urethral valve, renal dysplasia, renal failure, vesicoureteric reflux

## Abstract

There are not many studies on long term follow up of children following surgery for posterior urethral valve in India. This study was done to assess the growth and renal function of children who had completed five years after surgery for posterior urethral valve at our hospital. Thirty children were included in this study. They were assessed retrospectively for the age and pattern of presentation, time of surgery and outcome. Outcomes measured were stunting, renal failure (GFR, tubular functions) and bladder functions. Fifty per cent of children were symptomatic five years after surgery with enuresis, dribbling, polyuria and recurrent urinary tract infection (UTI). GFR was <60 ml/m/1.73 m^2^ in 33%. Growth failure, according to the World Health Organization (WHO) definition, was present in one-third of children. A low GFR was associated with growth failure. Poor bladder function evidenced by history of dribbling and significant residual urine was seen in one-third of patients. Residual hydronephrosis was seen in 74%. The most common presenting symptoms of PUV were poor urinary stream followed by recurrent UTI, poor weight gain, renal failure and abdominal mass. Eighty per cent of the study population had undergone surgery in infancy. Five years after surgery, 50% children were symptomatic; 30% had stunting. 33% had a GFR <60 ml/m/1.73 m^2^ and a significantly greater degree of stunting than those with GFR >60 ml/m/1.73 m^2^. Sonologically normal kidneys on follow-up were associated with a GFR above 60 ml/m/1.73 m^2^. Poor bladder function was present in 30% of the children. Univariate analysis showed that statistically significant risk factors for decline in GFR in this study are oligohydramnios and surgery beyond the neonatal period.

## Introduction

Posterior urethral valve (PUV) is the most common congenital anomaly in boys with an incidence of 1 in 8000 male births. It is the most common obstructive cause of end stage renal disease in children.

Vesicoureteric reflux, recurrent UTI, voiding dysfunction and late onset renal failure are the long term major problems in these children. There are a few long term outcome studies of children with PUV from India.[1–3] These studies mainly concentrate on the surgical aspects. The present study is aimed to assess the long term impact of PUV on renal function and the growth of these children.

## Materials and Methods

The study was conducted at SAT Hospital, Government Medical College, Thiruvananthapuram, between October 2006 and July 2007. Thirty children, with posterior urethral valve five years or more post surgery, were included in the study.

The details of children with regard to the age, presenting symptoms, serum creatinine, presence or absence of vesicoureteric reflux at surgery and surgical interventions done were obtained from records. On follow-up, they were assessed clinically. Weight and height were measured using standardized procedures. Biochemical analysis and ultrasound abdomen were done. Outcomes measured were stunting, renal failure (GFR, tubular functions) and bladder functions.

Stunting was classified according to the WHO norms and grading was done by Waterlows classification of height for age using NCHS standards[4] [Table 1].

**Table 1:** Classification of stunting

Grade of stunting	Percent of median height for age
Normal	>95
Mlid	90-94
Moderate	85-89
Severe	<85

Glomerular filtration rate (GFR) (ml/m/1.73 m^2^) was determined by applying the Schwartz formula:[5]

$$\mathrm{GFR}\;=\;\frac{k\;\times \mathrm{height}\;(\mathrm{cm})}{S.\;\mathrm{Creatinine}\;(\mathrm{mg}/\mathrm{dL})}$$

K is a constant. 0.55 for children and 0.7 for adolescents.

Based on GFR, according to the NKF-KDOQI guidelines, chronic kidney disease was classified into five stages.[6]

Tubular functions were assessed by the history of polyuria, urine specific gravity and presence of systemic acidosis. Polyuria was defined as urine output >2000ml per 1.73m^2^/24 hr or more than 3 ml/kg/day. Accurate measurement of 24 hours intake of fluids and quantity of urine passed was done to establish diagnosis of polyuria. Early morning sample of urine was tested on three consecutive days for specific gravity. The urine specific gravity of less than 1.010 and polyuria suggested abnormal tubular function.Acidosis was assessed by measurement of venous bicarbonate. The normal venous bicarbonate level was taken as 22 – 29 meq/L. The values below 22 meq/L were taken as evidence of acidosis.

Ultrasonography of abdomen was done to assess renal growth, asymmetry, presence of residual hydronephrosis and bladder residual volume. Bladder function was assessed by the history of dribbling and significant residual urine on ultrasound in those children without VUR.

### Statistical methods

Data was entered into Microsoft Excel for WINDOWS 2003 and analyzed by SPSS for Windows 11. For normally distributed variables mean and for variables not-normally distributed, median was calculated. For comparison between two groups, Chi–square test and Mann – Whitney ‘V’ tests were done for variables that are not-normally distributed. Univariate analysis was done to assess risk factors for decline in GFR.

## Results

Thirty children with PUV fulfilled the criteria and were analyzed. The age at presentation varied from antenatal detection to six years. About 46.6% of patients presented between 0-1 month, 36.6% between one month – one year and 16.8% between one to six years. The median age at presentation was three months. Primary surgery was done in the neonatal period in 33% children.

Of the 28 children who had antenatal ultrasound, 20 had normal USS and eight had antenatally detected hydronephrosis i.e. 28.6% of patients. Five out of the eight had associated oligohydramnios. All these five children had GFR <90ml/m/1.73 m^2^ at follow-up.

About 45% of patients had no VUR at diagnosis while 13.8% had unilateral VUR and 41.4% had bilateral VUR. The VUR in our study group was predominantly grades 4 and 5. Poor urinary stream was the commonest presentation (83%) followed by recurrent UTI (70%). The other symptoms were poor weight gain, renal failure and abdominal mass. Elevated serum creatinine was present at diagnosis in 63% of patients. 37% of them were oliguric and 57.9% had poor weight gain in infancy.

The age of the study population at follow-up ranged from 5-16 years with the mean of 7.78 years (2.6). 5 years after surgery, 50% of them were symptomatic. Enuresis was present in 47% patients, dribbling in 43%, polyuria in 40%, muscle cramps in 33%, recurrent UTI in 23% and bone pain in 13%. Of the 30 children included in our study, 33% had a GFR <60ml/m/1.73m^2^ at follow-up [Table 2].

**Table 2:** Staging of chronic kidney disease in children with PUV based on KDOQI classification

Stage	GFR	No.	%
1	90	4	13.3
2	60-89	16	53.4
3	30-59	4	13.3
4	15-29	5	16.6
5	<15	1	3.4

Using the WHO definition of stunting, growth failure was assessed. Stunting is defined by the WHO as a height for age more than a standard deviation of 2 below the median value of the reference population. Nine out of 30 patients i.e. 30% had growth failure. Of the six patients with GFR less than 30 ml/m/1.73 m^2^, 4 patients ie; 66.7% had stunting.

Using the NCHS reference standards for height and applying Waterlows classification, 43.4% had second degree stunting and 20% had third degree stunting. To study the relation between GFR and growth failure, the study population was divided into two groups – those with GFR <60 ml/m/1.73 m^2^ and those with GFR >60 ml/m/1.73 m^2^. Significant correlation was observed between low GFR and degree of stunting.

About 40% of children had polyuria. Venous bicarbonate levels were done in 26 patients. Of this, 15 patients had a bicarbonate <22 meq/L and 11 patients had a bicarbonate level >22 meq/L.

To study the relation between the presence of acidosis and GFR, the patients were divided into three groups: GFR <30 ml/m/1.73 m^2^, GFR 30-60 ml/m/1.73 m^2^ and GFR >60 ml/m/1.73 m^2^. In patients with GFR <30 ml/m/1.73 m^2^, the mean venous bicarbonate was 18.67 meq/L with a SD of 1.5, in those with GFR 30-60 ml/m/1.73 m^2^, the mean venous bicarbonate was 20.50 with a SD of 1.2 and in patients with GFR >60 ml/m/1.73 m^2^, the mean venous bicarbonate was 21.6 meq/L with a SD of 2. The results showed statistically significant difference.

Of the 10 patients with a GFR <60 ml/m/1.73 m^2^, 9 had acidosis with venous bicarbonate level <22 meq/L i.e.; 90% i.e. There was a statistically significant relation between the severity of acidosis and stage of CKD in this study. 88% (*n*=22) of the patients with GFR >30 ml/m/1.73 m^2^ in our study had urine specific gravity ≤1.010.

History of dribbling was present in 43% of children. USS abdomen showed significant residual urine in 30%. There was residual hydronephrosis in 74% patients – bilateral in 55.5% and unilateral in 18.5%. All 6 patients with GFR<30 ml/m/1.73 m^2^ had bilateral gross hydronephrosis and majority had significant residual urine – these two factors probably contributing to the more rapid deterioration of glomerular function. Those patients with a normal urinary tract on ultrasond abdomen at follow up had a GFR above 60 ml/m/1.73 m^2^.

Univariate analysis was done to assess the risk factors for decline in glomerular filtration rate [Table 3]. Statistically significant risk factors included oligamnios and surgery after the neonatal period. Antenatal detection, presence of vescicoureteral reflux and initial serum creatinine were not statistically significant. The “nadir creatinine” was not available from the records in many of these children and was not analyzed.

**Table 3:** Risk factors for decline in GFR (Univariate analysis)

Risk factors	GFR >60 (*n*=20)	GFR <60 (*n*=10)	*P*-value
Surgery beyond neonatal period	10	9	0.03*
Presence of antenatal hydronephrosis	7	1	0.11
Oligamnios	1	4	0.02*
S. creatinine at presentation >0.8 mg/dl	16	10	0.17
Presence of VUR	9	7	0.18

* Statistically significant

## Discussion

In the recent decades, the immediate outcome of boys with PUV has improved continuously with the development of early diagnostic and treatment modalities. However, there is a growing concern over the long term outcome of these children as 24 to 45% of them develop renal failure in childhood or adolescence. Unfavorable prognostic indicators include antenatal presentation before 24 weeks of intrauterine life, renal dysplasia, poor corticomedullary differentiation on ultrasonography, B/L vesicoureteric reflux (VUR) and persistence of high serum creatinine.

Analysis of the clinical presentation of 30 children with PUV showed that the most common symptom at presentation was poor urinary stream followed by recurrent UTI, poor weight gain, renal failure and abdominal mass. Median age at presentation was 3 months. In a study by Parkhouse *et al*. one-third of patients were detected between 0-1 month, one-third between one month and one year and one-third between one and six years.[7]

Eighty per cent of the study population had undergone surgery in infancy. By univariate analysis, children whose surgery was beyond 28 days had statistically significant risk of poor glomerular function on follow up. Hydronephrosis was detected antenatally in 28.6%. If the amniotic fluid volume is low, the outcome is poor with low GFR. Those with hydronephrosis and oligohydramnios had a poorer outcome than those without oligohydramnios.

About 55.2% children had VUR at diagnosis and VUR was bilateral in 41.4%. Study by Parkhouse *et al*. reported the occurrence of VUR to be 25%.[7] In a study by Roth *et al*. unilateral VUR was present in 30% and bilateral VUR in 50%.[8] In a review from CMC vellore VUR was present in the newborn period in 30%.[2]

Five years after surgery, 50% children were symptomatic. The major symptoms at follow-up were enuresis, dribbling and polyuria. But urodynamic studies could not be done due to lack of facilities for the same. In a study by Lal *et al*. 35% had symptomatic voiding dysfunction, the most common symptom being nocturnal enuresis with diurnal urgency and frequency on long term follow-up.[9] In the study by Connor *et al*. 19% patients had urinary incontinence on follow-up.[10] These symptoms are due to the poor concentrating ability of the renal tubules along with poor bladder compliance.

Glomerular filtration rate was decreased i.e. <90 ml/m/1.73 m^2^ in 86.7%, <60 ml/m/1.73 m^2^ in 33.3% and severe reduction of GFR i.e. <30 ml/m/1.73 m^2^ in 20% patients. The study by Parkhouse *et al*. reported poor outcome in one third of patients.[7] In a follow-up study of 46 children with PUV with a mean follow-up of 12.5 years, E Ylinen *et al*. reported that 30% had a GFR <60 ml/m/1.73 m^2^.[11]

About 30% of children in our study group had growth failure in the form of stunting according to WHO definition. Those with GFR <60 ml/m/1.73 m^2^ had a greater degree of growth failure than those with GFR >60 ml/m/1.73 m^2^ and the difference was statistically significant. In a study by Tejani *et al*. with a mean follow-up of nine years, growth failure was present in 40% of patients.[12] In the long term follow-up study from India by A N Gangopadhyaya height was below 50^th^ centile in 52% children.[1]

The severity of metabolic acidosis increased with greater decline in GFR. A statistically significant relation was present between the fall in GFR and acidosis. Poor bladder function was present in 30% of the children as evidenced by significant post void residual urine on ultrasound. This was also associated with low GFR. Statistically significant risk factors in this study for decline in GFR are oligamnios and surgery after the neonatal period. Ansari *et al*. also had similar observations. They have reported that children with PUV presenting after two years have higher risk of developing chronic renal insufficiency on long term follow-up.[3]

The presence of vescicoureteral reflux was not a risk factor for decline in GFR in our study. This is in contrast to the previous studies by Elisa *et al*.[11] and Ansari *et al*.[3] The “nadir creatinine” was not available from the records in many of these children and was not analyzed.

Antenatal detection, counseling of the couple regarding the poor outcome if there is oligohydramnios, early fulguration before 28 days, assessment of GFR before surgery, assessment of yearly GFR, renal growth, tubular functions, bladder functions, optimization of reno protective measures and surgical interventions as and when needed on follow-up are important in the management of all children with posterior urethral valve. Comprehensive care should be the rule by a team comprising pediatrician, pediatric surgeon and pediatric nephrologists for prompt diagnosis and management of upper and lower urinary tract of these children. This will go a long way in reno protection and delaying the occurrence of kidney failure in children with corrected PUV. It also helps in early planning of renal replacement therapies in children with progressive renal insufficiency.
